RETRACTED

# The Effect of Mobile Social Media Sharing Behavior on the Subjective Well-Being and Mental Health Regulation of Internet Users

**DOI:** 10.1155/2022/7573322

**Published:** 2022-09-27

**Authors:** Mingqing Lu, Qiangqiang Ma

**Affiliations:** ^1^Ideological and Political Theory Teaching and Research Department, Changchun Automobile Industry Institute, Changchun 130013, China; ^2^School of Marxism, Jilin University of Finance and Economics, Changchun 130117, China

## Abstract

Mobile Healthcare Social Media (MHSM) is an innovative combination of mobile devices and mobile communication technology. How can users shift from spontaneous to conscious cognitive mode, break their usage inertia, and actively adapt to the social structure of mobile health social media to improve information-sharing performance? This study uses adaptive structuring theory as the theoretical foundation to deeply analyze adaptive information-sharing behavior and its specific forms in the mHealth social media environment; it uses cognitive shift theory and social exchange theory as the theoretical framework to comprehensively explore the antecedent motivations of users engaging in adaptive information-sharing behavior and its posterior effects. Theoretically, it promotes the innovation and development of information-sharing behavior research and the further deepening of the application of adaptive structuring theory at the information behavior level. It is also conducive to bridging the digital divide and maximizing the value of health information resources. This paper takes 1000 survey data as the experimental data source for studying the influence of mobile social media sharing behavior on the subjective well-being and mental health regulation of Internet users and concludes that in practice, it is beneficial to optimize the design of information-sharing-related functions in mobile health social media, improve the effect of user information sharing in mobile health social media environment, and enhance the efficiency of information sharing so that mobile social media sharing behavior can better contribute to the subjective well-being and mental health regulation of Internet users. This paper has an obvious psychological adjustment effect on groups who use too much social media and can help them analyze why they are affected by some social media, thereby producing psychological effects.

## 1. Introduction

The widespread use of wireless devices such as smartphones and tablets has not only brought users a variety of ways to communicate information (e.g., text, voice, video, and geolocation) but also promoted the development and innovation of many mobile applications that meet the multiple needs of personal information services and bring convenience to people's daily lives. Mobile social media has become one of the most popular mobile applications, relying on the advantages of more timely content and faster response to extend personal activities to social networking services so that information can be accessed and shared anytime and anywhere [1]. Social media is defined as technologies and applications based on web- and user-generated content, whose manifestations include content sharing and relationship building, providing users with the opportunity to generate, share, receive, and comment on social content among multiple users through multisensory communication. Social media has changed the way people communicate, which also includes the communication, sharing, and dissemination of health information [2].

RETRACTED

The emergence of social media has allowed people to use the medium for their own and others' social interactions and information dissemination without the need to engage in real communicative activities [3]. International research on social media has reciprocally studied the profile of information dissemination on social media and its effects on social support, subjective well-being, and intimate relationships. Studies have shown that mobile media devices such as smartphones and tablets further contribute to the formation and development of microblogging dependence among college students, who mainly use Facebook to obtain information, entertain, and amuse themselves and maintain and expand their interpersonal relationships; and that older users who have used it for more than a year are more likely to become dependent on it, with the degree of dependence gradually deepening over time.

Happiness is a complex, multilevel psychological state formed by the interaction between psychological factors such as needs (including interests, motivations, and desires), cognition, emotions, and some external triggers and is an emotional-emotional state that arises when individual human needs are met and when ideals are realized [4]. Psychologists study people's well-being from the subjective feelings and position of the studied person and consider subjective well-being as an overall assessment of an individual's life situation according to self-defined criteria. The definition of subjective well-being differs from researcher to researcher, but researchers generally agree with Diener's definition, which considers subjective well-being as an overall assessment of an individual's quality of life based on self-determined criteria [5]. He defines happiness in terms of an individual's self-evaluation, emphasizing the individual's subjective experience and the individual's internal needs and perceptions of value under objective life conditions. The present study continues his definition of subjective well-being [6] and defines subjective well-being as “the overall evaluation of the quality of a person's life based on his or her subjective criteria.”

RETRACTED

## 2. Related Discourses

Currently, relatively little research has been conducted outside the globe directly on social media dependence, with studies focusing on reliance on specific items included in social media, such as Twitter and Facebook, and findings suggesting that the impact of reliance on these social media on people's lives includes both positive and negative aspects. International research on social media has been peer-to-peer, examining the profile of information dissemination on social media and its effects on social support, subjective well-being, and intimate relationships.

Di Domenico [7] et al. studied the use of social media in the United States and concluded that social media has changed the way people communicate in many ways. Vraga and Tully [8] showed that social media can lead to more social support and social skills for college students. Li [9] et al. studied the role of social media in romantic relationships and showed that the self-esteem shown in the use of social media has an impact on jealousy and happiness in romantic relationships, and that jealousy and happiness in individuals with low self-esteem are more influenced by social media. By studying the correlation between use and attachment styles and social skills, they found that individuals with high levels of anxiety used more frequently when feeling negative emotions or concerned about how others perceive them, whereas individuals with low levels of anxiety were less likely to use it. In addition, participants who scored high on social skills (social sensitivity, social expressiveness, and social control) tended to use them more and more intensively. Other researchers have examined the relationship between use and personality and have shown that there are significant personality differences between nonusers and frequent users of social software. Nonusers had a lower tendency to confide in themselves and masked narcissistic behavior, while frequent users scored higher on overt narcissistic behavior as well as on intimate feelings, suggesting that intimate feelings may extend to social networks, allowing such intimacy to be experienced both online and offline. Cao and Yu [10] developed the aneurysm scale to diagnose those who are over or even addicted to using, which has six factors: emergent behavior refers to manifestly obvious behaviors; tolerance refers to the level of tolerance; withdrawal refers to the bad feelings after nonuse; flat rate of a reuse after the relapse phase; conflict refers to moods that are filled with ambivalence; and mood change refers to changes in mood. The online interaction questionnaire for college students developed by Li et al. [11] consists of online interaction awareness, which refers to the awareness of online interaction. Network interaction social perception refers to the social information perceived about network interaction. Network interaction information communication refers to self-communication and others' communication of network interaction information. The negative outcome of network interaction refers to the bad outcome of the process of network interaction. Network interaction self-exposure and emotional experience refer to the self-study and self-recreation in network interaction, and network interaction recreation refers to playing games on the Internet.

RETRACTED

Various interpretations of the definition of social media exist in academia but reflect common connotations. Pee [12] considers social media to be characterized by participation, openness, communication, dialogue, community, and connectivity, and a new type of online media that gives users great space for participation and freedom of engagement. Pentina et al. [13] consider social media as a web application based on Web 2.0 technologies and ideologies that allow individual users to generate content and communicate online. Although slightly different in formulation, the essence of “consumer as producer” and “user-created content,” as well as the extension of social media (“blogs,” “microblogs,” and other media expressions), have been discussed. However, the essence of “consumers are producers” and “users create content,” as well as the extension of social media (blogs, microblogs, etc.) are more consistent. Compared with traditional media, social media breaks the “one-to-many” communication model, and users use online services in a participatory and collaborative manner. Social media is a product of the interplay between personal information space and public information space, and the use of social media facilitates a paradigm shift in the way people communicate, collaborate, create, and consume information. According to Lee and Jin [14], information behavior refers to “the sum of human behaviors associated with information sources and channels.” Seo et al. [15] consider information behavior as an integrated process of individual information seeking, information foraging, meaning construction, information searching, information organization, and information used around a single topic or multiple topics. Khan and Idris [16] define information behavior as “the activities that individuals engage in when they identify their information needs and seek, use, or transmit information in some way” using information needs as a research perspective.

RETRACTED

Moreno et al. [17] state that “information sharing is one of the dimensions of information use and is the process by which individuals acquire information and pass it on to others.” From the perspective of communication effects, information sharing is the activity of information providers to disseminate identified information to information seekers. From a behavioral perspective, Graham et al. [18] define information sharing in three dimensions: from a synergistic perspective information-sharing behavior is an activity in which information providers and information seekers jointly accomplish the transfer of certain information from the former to the latter; from a reciprocal perspective information-sharing behavior can be defined as the exchange of information between information providers and information seekers in collaboration to achieve their respective or common interests [19]; from socialization, in terms of reciprocity, information sharing can be defined as a collaborative exchange of information between information providers and information seekers to achieve their respective or common interests. This leads to a more comprehensive and three-dimensional definition of information sharing: information sharing is an information behavior in which information providers and information seekers with specific relational connections collaborate through information exchange to achieve individual or common interests. In the social media environment [20], users share information mainly by posting their ideas, information, and experiences through comments and messages to provide information sources for other users who are interested in learning or acquiring information.

## 3. The Impact of Mobile Social Media Sharing Behavior on Internet Users

### 3.1. The Influence of Mobile Social Media Sharing Behavior on Internet Users' Subjective Well-Being

Based on in-depth interviews to root out the factors influencing adaptive information-sharing behavior, six main categories influencing adaptive information-sharing behavior of mHealth social media users were identified, namely, new context, difference, intentional requirements, perceived risk [21], control beliefs, and personal traits, which were distilled from 14 subcategories, namely, others' use, technological environment change, and expectation inconsistency. The six main categories are distilled from the following 14 subcategories: use by others, changes in the technological environment, inconsistent expectations, (subjective) intentional requirements, (objective) intentional requirements [22], information risk, operational risk, time/effort risk, social risk, competence, facilitation, personality traits, mental state, and demographic characteristics. In this chapter, based on the rooted analysis in chapter 3, we will explore and hypothesize the influencing factors of adaptive information-sharing behavior of mHealth social media users concerning the sources of subcategories and the reference number (i.e., the number of free nodes) and construct a research model of adaptive information sharing influences by combining relevant studies in cognitive shift theory, social exchange theory, control beliefs, and emotions [23].

RETRACTED

This study uses cognitive shift theory as the main research perspective to explore the triggering conditions of adaptive information-sharing behavior. Adaptive IT use research falls within the field of technology acceptance and use research, and existing research identifies technology environment factors, individual factors, and social factors as important antecedent variables of technology acceptance and use. The technological environment represents opportunities and constraints in this study setting that may facilitate or hinder the achievement of an individual's goals. Considering the social nature of mHealth social media, postadoption behavior should be fully considered in the evaluation of exchange relationships between users. Social exchange theory emphasizes the exchange relationships between social actors (individuals and groups organizations) and provides a research perspective on the interaction between individuals and the social environment. Finally, the adaptive information-sharing behavior of mHealth social media users is a cognitive and behavioral breakthrough based on daily, repetitive, and customary use; and therefore, individuals need to have sufficient resources required for IT innovation such as competence, experience, external support, and positive emotions to support users' exploration of the system. In summary, this study constructs a model of factors influencing adaptive information behavior among mHealth social media users based on three main scenarios of cognitive shift and considering the role of perceived risk as a hindrance to adaptive information-sharing behavior and the role of control beliefs and positive emotions as a facilitator of adaptive information behavior.

#### 3.1.1. Social Media Sharing Behavior Model Construction

An interview rooting analysis of adaptive information sharing among health social media users found that the dynamic evolution of the social structure embedded in mHealth social media offers the possibility of diverse user use, with information sharing as a goal-oriented approach and to improve the effectiveness and enhance the efficiency of information sharing in practice, users can fully exploit the potential of existing system functions and explore more ways of implementing system functions. So as to build a model of social media sharing behavior. Its theoretical formula is

(1) $$\begin{array}{c} M=\frac{\Delta y}{\Delta x}.\frac{\partial^{2}\Omega }{\partial v^{2}}. \end{array}$$

The rapid development of mobile health social media and the diversity and complexity of users' health information needs have brought about adaptive use of system functions by users. Based on the results of the above social structure profiling and rooting analysis, this section summarizes and concludes the different ways of users' adaptive use of mHealth social media for information sharing, constructs a higher-order model of adaptive information-sharing behavior, and reveals the specific performance differences of users' adaptive information behavior. The developmental use and explorative use are pointed out as the ways of using information systems in the internalization/integration stage, with the developmental system use being the use related to short-term task performance and the explorative use being linked to long-term task performance. The conceptualization of the technology use phase is summarized as shown in Figure 1.

RETRACTED

#### 3.1.2. Second-Order Model Construction of Social Media Sharing Behavior

Adaptive structuring theory assumes that regardless of the features designed in the system, users can tune the technology effects, adopt and debug to adapt the system to their needs, and that there are multiple ways to resist or not use that have different effects on the technology effects. The implementation of the technology is determined by the adaptation and usage patterns of the users. This suggests that users can often engage in change adaptation practices. The formula principle is

(2) $$\begin{array}{c} N=\overset{n}{\underset{i=1}{\sum }}X_{i}^{2}+\frac{1}{n}\overset{n}{\underset{i=1}{\sum }}{\left(X_{i}-\bar{X}\right)}^{2}. \end{array}$$

Change adaptation is best described as a modification of the built-in functionality of the technology that helps people do their jobs. According to adaptive structuration theory, technology contains both predetermined and realistic social structures and deviations between the two social structures depend on how individuals/organizations use the technology appropriately or select certain structures to meet situational needs or engage in universal practices. Adaptive structuring theory suggests two different ways of adapting: (i) adopting the technology faithfully, meaning that the user uses the technology in a way that is consistent with the spirit of the technology (e.g., the design intent of the technology developer); and (ii) adopting the technology disloyally, meaning that the technology is used in a way that is inconsistent with or contrary to the design intent of the technology. Of course, the set of spirits embedded in the technology is not exclusively the designer's intent; these designer's intents are a reflection of the technology's embedded set of spirits. Existing research on information use based on adaptive structuring theory has focused on two dimensions: loyal adaptation and disloyal adaptation. A study of adaptive information system use based on modifying IT content and modifying the spirit embedded in IT (designer intent) argues that modifying the content of in-use features is about which specific features to use and modifying the spirit of in-use features is about how to use those features, proposing a higher-order model of adaptive system use that can better derive the effect of mobile social media sharing behavior on Internet users' subjective well-being, as Figure 2 shows.

RETRACTED

### 3.2. The Influence of Mobile Social Media Sharing Behavior on the Regulation of Internet Users' Mental Health

The concept of Information Seeking Anxiety (ISA) emerged earlier in 2012, arguing that with the continuous development of network technology and the ever-changing information environment, people's access to information has become diversified, and multimedia and information seeking anxiety does not only appear in the category of early library anxiety. In today's mobile social media environment, information seeking anxiety is not only in the context of early library anxiety. When external information is input into the brain, the human brain has a high-level center to synthesize, analyze, and judge. The brain will absorb a large part of the information. If it cannot absorb it, it will feel anxious.

In today's mobile social media environment, users' information seeking anxiety is also characterized as follows: (1) mobile social media is characterized by a large flow of information and fast turnover based on which users have more information needs in immediate situations, and if they engage in information seeking behavior, they are likely to face potential information seeking anxiety in this process. This kind of information seeking anxiety triggered by immediate situations is difficult to predict and control. (2) There are numerous types of mobile social media, and the functions and features of different platforms are naturally different. The same user's preference for different platforms and the degree of praise and criticism of the same platform by different users can affect the efficiency and results of information seeking. Therefore, when discussing the information seeking anxiety under mobile social media, it is not only different from person to person and platform to platform but also the degree of fit between users and platforms should be considered. In the face of this uneven quality or even false information, users still need to identify the authenticity and credibility of the information after the information search “results” are presented. This increases the cost of eliminating information seeking anxiety for users.

RETRACTED

#### 3.2.1. Mobile Social Media Increases Information Anxiety of Internet Users

Research on fear of missing out dates back to 2013 and is recognized as the first time researchers have explored the concept from an academic perspective. Missing out anxiety is the worry and apprehension that occurs when a user loses contact with others, is absent, or misses out on an experience that others might otherwise receive or enjoy. When experiencing loss anxiety, people show a strong desire for information and access to the behavior of others and continue to collect such information, and users' internal appeals when experiencing loss anxiety, i.e., when faced with loss anxiety, are immersed in a psychological need to connect with others, gain attention, and fit in.

Users in the mobile social media environment are often faced with registration, link sharing, authentication, and other uploads involving personally identifiable information. Well-known social platforms at home and abroad have a large registration base and store a large amount of personal data, and these social platforms have become the main targets of cyber hacking attacks. Traditional cyber attacks and risks are spreading to IoT and smart devices with an increased risk of data leakage.

Anxiety about missing information, also known as fear of missing out, refers to a diffuse compound emotional experience that is dominated by anxiety and accompanied by negative feelings such as fear, loss, worry, and depression resulting from missing some possible important information or novel events. The network brings rich information resources to users, but with the continuous development of ICT, information organization forms become diversified, and the number of information is growing exponentially, showing an overload situation. With the continuous integration of social networks and technologies, new types of overload have entered people's lives, mainly including redundancy and falsity of information, involuntary expansion of social networks (e.g., pushing, and prompting), and rapid changes in the technical functions of social networks.

RETRACTED

#### 3.2.2. Model Construction of Mobile Social Media Users' Heart Health Regulation

The theoretical model selected for this study is the Stressor-Strain-Outcome Theory Model (Stressor-Outcome Model). This model is widely used in studies where stressors are used as an independent variables, and researchers can explore the influence of stressors on mediating variables and possible behavioral consequences through different path analyses and is considered a classical analytical tool for stressor influence mechanisms in the field of management psychology. In the SSO model, emotional states can also be used as mediating variables to further explore the possible consequences for users after strain stress In the SSO model, emotional states can also be used as mediating variables to further explore the psychological or behavioral consequences that may arise after a user is stressed.

In the SSO model, emotional states can also be used as mediating variables to further explore the possible psychological or behavioral consequences of users after strain, the Stressor-Strain process, and in addition, a preliminary attempt was made in terms of the possible behavioral consequences of users' information anxiety (i.e., outcome analysis). Thus, the empirical research path of this paper and the SSO model are highly consistent. Therefore, the SSO model is chosen for the follow-up study. The study path is shown in Figure 3.

## 4. Experimental Design

After the initial construction of the SSO model of user information anxiety in the mobile social media environment, the hypotheses in the model still need to be verified with the support of data analysis to test and revise the model until the final theoretical model is formed. This paper adopts the questionnaire survey method to conduct an empirical study on Internet users, and the sample selection is based on the following considerations: whether the sample selection is representative, whether the sample data is accessible, and whether the sample selection is random. (1) Students can be seen on all major social media platforms. Therefore, the attention to student groups has corresponding research value. (2) The student group is relatively concentrated and shows high enthusiasm in participating in various questionnaires, and can accept and complete the questionnaires independently and patiently. Therefore, the sample data has high accessibility.

## 5. Analysis of Results

### 5.1. Analysis of Experimental Results on the Influence of Mobile Social Media Sharing Behavior on Internet Users' Subjective Well-Being

In this paper, the experiments use the Structural Equation Modeling (SEM) technique to verify the model and model hypotheses of the factors influencing the information-sharing behavior of mobile health social media users based on theoretical literature research and interview content rooting analysis. On the issue of the sample size of the questionnaire, “SEM is suitable for the analysis of large sample data, and the larger the number of samples taken, the better the stability of SEM statistical analysis and the applicability of various indicators. Usually, more than 200 samples can be called a medium-sized sample, if you want to pursue better stability of SEM analysis results, the number of samples subjected to the best is 200 or more,” so this experiment selected 1000 samples of data. Its use of SEM techniques and traditional analysis techniques appeared to be significantly different in efficiency, and its experimental results are shown in Figure 4.

RETRACTED

Reliability analysis is used to measure whether the results of the sample responses are reliable and whether the sample has truly answered the scale-type questions. Reliability analysis measures only the quantitative data, i.e., the third part of the questionnaire. The Cronbach alpha coefficient is usually used as a measure. If the coefficient is above 0.8, the reliability of the questionnaire is very good; if the coefficient is between 0.7 and 0.8, the reliability of the item is good and can enter the formal survey; if the coefficient is above 0.6, the questionnaire as a whole has a certain research necessity, but the scale scoring questions involved in the questionnaire need to be revised appropriately. The effect of mobile social media sharing behavior on the subjective well-being of Internet users is different from those who do not share their lives online, and the comparison of their well-being is shown in Figure 5.

### 5.2. Analysis of Experimental Results on the Psychological Impact of Mobile Social Media Sharing Behavior on Internet Users

When we experimented on the psychological effects of mobile social media sharing behavior on Internet users, we put the compulsive symptom factor, paranoia factor, hostility factor, interpersonal tension and sensitivity factor, depression factor, anxiety factor, learning stress factor, maladjustment factor, emotional imbalance, psychological imbalance factor, achievement goal pressure, external environmental pressure, frustration pressure, competitive pressure and expression inhibition, cognitive reappraisal, etc. The common method bias test refers to the fact that all data come from the same subject, and the same testing environment and some characteristics of the topic itself affect the relationship between the independent and dependent variables, which in turn will affect the results of the study. In study 2, the data of several variables are provided by the same research subject, and the questionnaire method is mainly used, and in study 2, the same questionnaire method is used. Harman's one-way test was used to test for common method bias. The experimental results of the impact of mobile social media sharing behavior on various aspects of mental health are shown in Figure 6.

RETRACTED

For Internet users, whether this behavior leads to the existence of mental health differences on Internet users, the presence of sharing behavior on mobile social media had significant standardized direct and standardized indirect effects on mental health. The results indicate that cognitive reassessment plays a partially mediating effect between academic stress and mental health, where the mediating effect size is −0.195 × (−0.308) = 0.06, and its comparative efficiency is shown in Figure 7.

## 6. Conclusion

In this study, we took Internet users of different ages as the research subjects and explored the impact of this behavior on the mental health of Internet users and the impact on their well-being from the perspective of whether they share their lives and opinions on mobile social media while studying the partial mediating role of emotion regulation between the two. Finally, through data analysis, the hypotheses in the previous paper were verified, most of them were valid, and only a few of them were partially valid, which indicated that the hypotheses of this study were well-confirmed, and the research results were better. The current social media dependence of Internet users is at a moderate to a high level, with large differences among different individuals. There were no significant differences in total social media dependence scores by grade level, and there were significant differences in compulsive behaviors and emotions by grade level. In conclusion, the perspective of sharing one's life and opinions on mobile social media can enhance the well-being of Internet users and regulate their psychological problems, but still within the appropriate context. This research should pay more attention to the efficiency of psychological adjustment and how to have specific adjustment measures in the follow-up.

## Figures and Tables

**Figure 1:** IT implementation process and usage stages.

**Figure 2:** On the construction of the higher-order model of the adaptive information system.

**Figure 3:** Stressor-Strain-Outcome theoretical model.

**Figure 4:** Efficiency differences between SEM techniques and traditional analysis techniques.

RETRACTED

**Figure 5:** Impact of mobile social media sharing behavior on Internet users' happiness.

**Figure 6:** Impact of mobile social media sharing behavior on various aspects of mental health.

**Figure 7:** The presence or absence of sharing behavior on mobile social media on mental health.

## Data Availability

The data used to support the findings of this study are available from the corresponding author upon request.
